The article "Removal of high density Gaussian noise in compressed sensing MRI reconstruction through modified total variation image denoising method" was retracted in 2025. Reasons: unreliable results or conclusions; concerns about the authorship.

# Removal of high density Gaussian noise in compressed sensing MRI reconstruction through modified total variation image denoising method^☆^

**DOI:** 10.1016/j.heliyon.2020.e03680

**Published:** 2020-03-30

**Authors:** Yonggui Zhu, Weiheng Shen, Fanqiang Cheng, Cong Jin, Gang Cao

**Affiliations:** a School of Data Science and Media Intelligence, Communication University of China, Beijing, 100024, China; b School of Information and Communication Engineering, Communication University of China, Beijing, 100024, China; c School of Computer Science and Cybersecurity, Communication University of China, Beijing, 100024, China

**Keywords:** Medical imaging, Mathematics, Total variation denoising, *K*-space data, MRI reconstruction, Compressed sensing

## Abstract

A modified total variation MRI image denoising method is proposed in this paper. First, the proposed method removes the noise in *K*-space in compressed sensing MRI reconstruction. Then, the removed *K*-space data is used as a partial frequency observation in compressed sensing MRI model. The proposed method shows better results than RecPF method, LDP method, TVCMRI method, and FCSA method in sparse MRI reconstruction. The proposed method is tested against Shepp-Logan phantom and real MR images corrupted by noise of different intensity level, and it gives better Signal-to-Noise Ratio (SNR), the relative error (ReErr), and the structural similarity (SSIM) than RecPF, LDP, TVCMRI, and FCSA.

## 1 Introduction

There are many methods that are able to accurately reconstruct the Magnetic Resonance images from highly undersampled *K*-space data in compressed sensing MRI (CS-MRI) field [1], [2], [3], [4], [5], [6]. Let N=m×n. Suppose $u\in R^{N}$ is a vector formed by stacking the columns of a two-dimensional MRI array $\left(u_{i,j}\right)$, i=1,…,m, j=1,…,n. The sparse MRI reconstruction model using wavelet and total variation is as follows:

(1) $$\min_{u}\frac{1}{2}{∥PFu-b∥}_{2}^{2}+\lambda {∥\psi u∥}_{1}+\alpha TV(u),$$

where *λ* and *α* are positive parameters, *ψ* is a wavelet transform, TV(u) is the total variation of *u*, *PF* is a partial Fourier matrix, $P\in R^{M\times N}$ consists of M≪N rows of the identity matrix, *F* is a two-dimensional discrete Fourier matrix that can be obtained by the Kronecker tensor product of two one-dimensional discrete Fourier matrices, and *b* is an observed *K*-space vector that is contaminated by Gaussian noise with standard deviation *σ*. The existing MRI reconstruction methods [1], [2], [3], [4] mainly consider the case of low-density noise for observed *K*-space data *b*. In fact, MRI acquisition may result in corrupted *K*-space data with high-density noise. The removal of high-density noise in MRI images and image processing have been studied by many researchers [7], [8], [9], [10], [11], [12]. For example, high impulse noise intensity for MRI images can be removed by adaptive median and fixed weighted mean filter (AMFWMF) [11]. The removal of high-density noise in corrupted images can be done by the boundary discriminative noise detection (BDND) [12] and improved boundary discriminative noise detection filter (IBDND) [8]. The high salt and pepper noise in degraded images can be removed by the modified decision based unsymmetric trimmed median filter [7]. However, to our knowledge, there is little research for the removal of high-density noise in frequency domain, i.e., *K*-space in compressed sensing MRI. In this paper, we focus on the removal of high-density Gaussian noise for observed *K*-space data in compressed sensing MRI. The proposed denoising method in this paper shows better performance than the existing methods in [1], [2], [3], [4]. In recent years, there are still many compressive sensing reconstruction methods. For example, Y. Liu et al. [13] exploited the available structure information to do biomedical signal reconstruction based compressive sensing methods. B. Trémoulhéac et al. [14] used low-rank and sparse prior information to reconstruct dynamic MR image from undersampled (k,t)-space. In [15], 2-D omnidirectional total variation (OTV) regularization is used to reconstruct hybrid CS-MRI with periodic time-variant subsampling. J. Yao et al. [16] proposed an efficient algorithm for dynamic MRI reconstruction method via low-rank and total variation regularization. Based on nuclear norm and total variation regularization, Z. Zhu et al. [17] developed a primal-dual algorithm to reconstruct dynamic magnetic resonance images. In particular, some important references [18], [19], [20] are tightly related to MRI denoising and reconstruction.

The article "Removal of high density Gaussian noise in compressed sensing MRI reconstruction through modified total variation image denoising method" was retracted in 2025. Reasons: unreliable results or conclusions; concerns about the authorship.

The rest of the paper is organized as follows. Section 2 presents a modified total variation MRI image denoising method. In Section 3, a new effective algorithm to solve problem (1) with high noise level is proposed. In Section 4, we use Shepp-Logan phantom and real MR images in numerical experiments to demonstrate effectiveness of our method in presence of high level noise for MRI reconstruction. Finally, some concluding remarks are presented in Section 5.

## 2 A modified total variation MRI image denoising method

The term ${∥PFu-b∥}_{2}^{2}$ in (1) is equal to ${∥Real(PFu)-Real(b)∥}_{2}^{2}+{∥Imag(PFu)-Imag(b)∥}_{2}^{2}$, in which Real(⋅) and Imag(⋅) represent the real and imaginary part of (⋅). Thus, corresponding to (1), we have

(2) $$\min_{u}\frac{1}{2}{∥Real(PFu)-Real(b)∥}_{2}^{2}+\frac{1}{2}{∥Imag(PFu)-Imag(b)∥}_{2}^{2}\;\;+\lambda {∥\psi u∥}_{1}+\alpha TV(u).$$

Let $Real(PFu)=v_{1}$, $Imag(PFu)=v_{2}$, $Real(b)=b_{1}$, $Imag(b)=b_{2}$, (2) can be formulated as

(3) $$\min_{u}\frac{1}{2}{∥v_{1}-b_{1}∥}_{2}^{2}+\frac{1}{2}{∥v_{2}-b_{2}∥}_{2}^{2}+\lambda {∥\psi u∥}_{1}+\alpha TV(u).$$

For (3), first solve two denoising problems:

(4) $$v_{1}^{⁎}=\arg\min_{v_{1}}{∥v_{1}-b_{1}∥}_{2}^{2}+2\mu TV(v_{1}),$$

(5) $$v_{2}^{⁎}=\arg\min_{v_{2}}{∥v_{2}-b_{2}∥}_{2}^{2}+2\mu TV(v_{2}).$$

In which, *μ* is positive parameter. Both (4) and (5) are *K*-space data denoising models given by Rudin, Osher and Fatemi [21]. It is well known that TV regularizier can better recover piecewise smooth signals with preserving sharp edges or boundaries. Next, let $b^{\prime }=v_{1}^{⁎}+v_{2}^{⁎}i$, *i* is the imaginary unit, i.e. $\sqrt{-1}$, solve the reconstruction problem as

(6) $$\min_{u}\frac{1}{2}{∥PFu-b^{\prime }∥}_{2}^{2}+\lambda {∥\psi u∥}_{1}+\alpha TV(u).$$

Compared with (1), $b^{\prime }$ in (6) is denoised *K*-space data corresponding to the previous observed noisy *b*. Therefore after solving (4) and (5), the reconstruction quality of MRI image by solving (6) is better than directly solving (1). In section 4, we will validate this result with numerical experiments. Problems (4) and (5) are the total variation models introduced by Rudin-Osher and Fatemi (ROF) in [21]. They can be solved by fast gradient-based algorithms introduced by A. Beck and M. Teboulle [22]. In the next section, we will give fast gradient-based algorithm for solving (4) and (5).

## 3 A new effective algorithm to solve problem (1)

For both problems (4) and (5), we consider the unconstrained denoising problem as the following.

(7) $$\min_{x\in R^{m\times n}}{∥\text{x}-B∥}_{F}^{2}+2\mu TV(\text{x}).$$

In which, *TV* can be chosen as the isotropic $TV_{I}$ and $l_{1}$-based anisotropic $TV_{l_{1}}$ given in [22].

Before construct a dual of problem (7) for $TV=TV_{I}$, following [22], we give some notation as follows.

• P is matrix-pair (p, q) where $\text{p}\in R^{(m-1)\times n}$ and $\text{q}\in R^{m\times (n-1)}$ that satisfy

$$p_{i,j}^{2}+q_{i,j}^{2}\leq 1,\;\;i=1,\ldots ,m-1,j=1,\ldots ,n-1$$

$$|p_{i,n}|\leq 1,\;\;i=1,\ldots ,m-1$$

$$|q_{m,j}|\leq 1,\;\;j=1,\ldots ,n-1.$$

• The operation $\text{L}:R^{(m-1)\times n}\times R^{m\times (n-1)}⟶R^{m\times n}$ is defined by

$$\text{L}{\left(\text{p, q}\right)}_{i,j}=p_{i,j}+q_{i,j}-p_{i-1,j}-q_{i,j-1},\;\;i=1,\ldots ,m,j=1,\ldots ,n$$

where $p_{0,j}=p_{m,j}=q_{i,0}=q_{i,n}=0$ for i=1,…,m and j=1,…,n.

• The adjoint of L is

$${\text{L}}^{T}(x)=(\text{p, q})$$

where $\text{p}\in R^{(m-1)\times n}$ and $\text{q}\in R^{m\times (n-1)}$ are matrices

$$p_{i,j}=x_{i,j}-x_{i+1,j},\;\;i=1,\ldots ,m-1,j=1,\ldots ,n$$

$$q_{i,j}=x_{i,j}-x_{i,j+1},\;\;i=1,\ldots ,m,j=1,\ldots ,n-1.$$

Proposition 3.1 *Let* (p,q)∈P *be the solution of the following problem*

(8) $$\min_{(p,q)\in P}h(p,q)\equiv {\left\|B-\mu L(p,q)\right\|}_{F}^{2}.$$

*Then the optimal solution of* (7) *is*

(9) x=B−μL(p,q).

The article "Removal of high density Gaussian noise in compressed sensing MRI reconstruction through modified total variation image denoising method" was retracted in 2025. Reasons: unreliable results or conclusions; concerns about the authorship.

The proof can be easily obtained by the proof of Proposition 4.1 when $H_{C}(\text{x})=\text{0}$ in [22].

Remark 3.1 The difference in problem (7) corresponding to the case $TV=TV_{l_{1}}$ is that the minimization is done over the set ${\text{P}}_{1}$ of matrices (p, q) where $\text{p}\in R^{(m-1)\times n}$ and $\text{q}\in R^{m\times (n-1)}$ satisfying

$$|p_{i,j}|\leq 1,\;\;i=1,\ldots ,m-1,\;\;j=1,\ldots ,n$$

$$|q_{i,j}|\leq 1,\;\;i=1,\ldots ,m,\;\;j=1,\ldots ,n-1.$$

Lemma 3.1 *Let* L(h) *be the Lipschitz constant of the gradient of the objective function h given in* (8)*. Then*

(10) $$L(h)\leq 16\mu^{2}.$$

Proof Since

$$\nabla h(\text{p, q})=-2\mu {\text{L}}^{T}(B-\mu \text{L}(\text{p, q})),$$

we have

$$\left\|\nabla h({\text{p}}_{1},{\text{q}}_{1})-\nabla h({\text{p}}_{2},{\text{q}}_{2})\|=2\mu \|{\text{L}}^{T}(B-\mu \text{L}({\text{p}}_{1},{\text{q}}_{1}))-{\text{L}}^{T}(B-\mu \text{L}({\text{p}}_{2},{\text{q}}_{2}))\right\|$$

$$\leq 2\mu \|{\text{L}}^{T}\|\|(B-\mu \text{L}({\text{p}}_{1},{\text{q}}_{1}))-(B-\mu \text{L}({\text{p}}_{2},{\text{q}}_{2}))\|$$

$$=2\mu^{2}\|{\text{L}}^{T}\|\cdot \|\text{L}({\text{p}}_{1},{\text{q}}_{1})-\text{L}({\text{p}}_{2},{\text{q}}_{2})\|$$

$$\leq 2\mu^{2}\|{\text{L}}^{T}\|\cdot \|\text{L}\|\cdot \|({\text{p}}_{1},{\text{q}}_{1})-({\text{p}}_{2},{\text{q}}_{2})\|$$

$$=2\mu^{2}{\left\|{\text{L}}^{T}\right\|}^{2}\cdot \|({\text{p}}_{1},{\text{q}}_{1})-({\text{p}}_{2},{\text{q}}_{2})\|.$$

For the operator ${\text{L}}^{T}$, we have

$${\left\|{\text{L}}^{T}(\text{x})\right\|}^{2}=\sum_{i=1}^{m-1}\sum_{j=1}^{n}{\left(x_{i,j}-x_{i+1,j}\right)}^{2}+\sum_{i=1}^{m}\sum_{j=1}^{n-1}{\left(x_{i,j}-x_{i,j+1}\right)}^{2}\leq 8\sum_{i=1}^{m}\sum_{j=1}^{n}x_{i,j}^{2}.$$

Therefore

$$\left\|{\text{L}}^{T}(\text{x})\|\leq \sqrt{8}\|\text{x}\right\|$$

meaning that $\|{\text{L}}^{T}\|\leq \sqrt{8}$. Thus, we obtain $L(h)\leq 16\mu^{2}$. The problem (8) can be solved by using Gradient Projection Method (GPM) that is formulated as

$$({\text{p}}_{k},\;{\text{q}}_{k})=P_{\text{P}}\left[({\text{p}}_{k-1},{\text{q}}_{k-1})-t_{k}\nabla h({\text{p}}_{k-1},{\text{q}}_{k-1})\right]$$

where $t_{k}$ is the stepsize chosen as the reciprocal of the upper bound on the Lipschtz constant, i.e., $\frac{1}{16\mu^{2}}$. Thus, the algorithm for solving the problem (7) can be described as follows.

The article "Removal of high density Gaussian noise in compressed sensing MRI reconstruction through modified total variation image denoising method" was retracted in 2025. Reasons: unreliable results or conclusions; concerns about the authorship.

Algorithm 1 **Input** B,μ and *K* (Maximum Number of Iterations)

**Output x**⁎ – An optimal solution of (7)

**Initialization** $({\text{p}}_{0},{\text{q}}_{0})=\left({\text{0}}_{(m-1)\times n},{\text{0}}_{m\times (n-1)}\right)$

**For** k=1,…,K **do**

$({\text{p}}_{k},{\text{q}}_{k})=P_{\text{P}}\left[({\text{p}}_{k-1},{\text{q}}_{k-1})+\frac{1}{8\mu }{\text{L}}^{T}(B-\mu \text{L}({\text{p}}_{k-1},{\text{q}}_{k-1}))\right]$

**End do**

**Set** ${\text{x}}^{⁎}=B-\mu \text{L}({\text{p}}_{K},{\text{q}}_{K})$

The above method has the rate of convergence of O(1/k) being proven in [22]. In order to improve the complexity result of Algorithm 1, the accelerated gradient-like method with an $O(1/k^{2})$ complexity result is used to solve the dual problem (8). The gradient-like method with the rate of convergence of $O(1/k^{2})$ was introduced by Nesterov in 1983 [23]. Following [22], now we give the Fast Gradient Projection Method (FGPM) on the unconstrained problem (7) as follows.

Algorithm 2 **Input** B,μ and *K* (Maximum Number of Iterations)

**Output** ${\text{x}}^{⁎}$ – An optimal solution of (7)

**Initialization** $({\text{r}}_{1},{\text{s}}_{1})=({\text{p}}_{0},{\text{q}}_{0})=\left({\text{0}}_{(m-1)\times n},{\text{0}}_{m\times (n-1)}\right),\;t_{1}=1$.

**For** k=1,…,K **do**

$({\text{p}}_{k},\;{\text{q}}_{k})=P_{\text{P}}\left[({\text{r}}_{k},{\text{s}}_{k})+\frac{1}{8\mu }{\text{L}}^{T}(B-\mu \text{L}({\text{r}}_{k},{\text{s}}_{k}))\right]$

$t_{k+1}=\frac{1+\sqrt{1+4t_{k}^{2}}}{2}$

$\left({\text{r}}_{k+1},{\text{s}}_{k+1})=({\text{p}}_{k},\;{\text{q}}_{k})+\left(\frac{t_{k}-1}{t_{k+1}}\right)({\text{p}}_{k}-{\text{p}}_{k-1},{\text{q}}_{k}-{\text{q}}_{k-1}\right)$.

**End do**

**Set** ${\text{x}}^{⁎}=B-\mu \text{L}({\text{p}}_{K},{\text{q}}_{K})$

After having the fast method to solve the problem (7), we can obtain a new effective algorithm to solve the original problem (1) as follows.

Algorithm 3 **Input** *b*− observed *K*-space data

**Step 1** $b_{1}⟵Real(b),\;\;b_{2}⟵Imag(b)$

**Step 2** Use Algorithm 2 to solve

$$v_{1}^{⁎}=\arg\min_{v_{1}}{∥v_{1}-b_{1}∥}_{2}^{2}+2\mu TV(v_{1})\;\;\text{and}$$

$$v_{2}^{⁎}=\arg\min_{v_{2}}{∥v_{2}-b_{2}∥}_{2}^{2}+2\mu TV(v_{2})$$

**Step 3** $b^{\prime }⟵v_{1}^{⁎}+\sqrt{-1}v_{2}^{⁎}$

**Step 4** Using the direct reconstruction algorithm to solve minimization problem

(11) $$u^{⁎}=\arg\min_{u}\frac{1}{2}{∥PFu-b^{\prime }∥}_{2}^{2}+\lambda {∥\psi u∥}_{1}+\alpha TV(u)$$

**Output** the optimal solution $u^{⁎}$

The direct reconstruction algorithm is the existed algorithm [1], [2], [3], [4]. The time complexity for Algorithm 3 is equal to the summation of Algorithm 2 and the existed algorithm. According to [22], we know that the fast gradient projection method is converged. Thus Algorithm 2 for solving two minimization problems in Step 2 has also converged. In addition, the existing direct reconstruction methods [1], [2], [3], [4] are also converged, so Algorithm 3 given by us is converged. Solving the problem (1) by Algorithm 3 has the better effect of denoising than directly solving the problem (1). The reason is that $b^{\prime }$ in (11) is the denoised result of *b* in (1). In the next section, using numerical experiments will show that Algorithm 3 has better denoising results than the existed direct reconstruction methods [1], [2], [3], [4], in particular, for the case of high level noise.

The article "Removal of high density Gaussian noise in compressed sensing MRI reconstruction through modified total variation image denoising method" was retracted in 2025. Reasons: unreliable results or conclusions; concerns about the authorship.

## 4 Numerical experiments

In this section, we evaluate the performance of Algorithm 3 in solving the problem (1) for CS-MRI. The signal to noise ratio (SNR), relative error (ReErr), and the structural similarity (SSIM) given in [24] are used to measure the quality of the reconstructed images. The signal-to-noise ratio (SNR) is defined as

(12) $$\text{SNR}=20\log10\left(\frac{{\left\|u_{o}\right\|}_{2}}{{\left\|u_{o}-u\right\|}_{2}}\right),$$

and the relative error (ReErr) is given as

(13) $$\text{ReErr}=\frac{{\left\|u-u_{o}\right\|}_{2}^{2}}{{\left\|u_{o}\right\|}_{2}^{2}},$$

where *u* and $u_{o}$ denote the reconstructed and original images, respectively.

We do tests on four images: a 256×256 Shepp-Logan phantom, a 256×256 brain image, a 220×220 chest image, and 210×210 brain image. All data are chosen according to the references [1], [2], [3], [4] in order to do comparison between the proposed method and other methods. In all tests, we add Gaussian noise for both the real and the imaginary parts of Fourier coefficients in sampling mask. For Shepp-Logan phantom shown in Fig. 1(a), we consider 66 radial lines in the frequency space with sampling ratio 26.85% shown in Fig. (b). And the additive noise has a mean zero and high level deviation 0.1. In the reconstruction test using Algorithm 3, we assume μ=0.02. Fig. 2 (a) and (b) show the reconstructed results by the proposed method and RecPF in [3]. The SNR, ReErr, and SSIM corresponding to the proposed method are 13.3147 dB, 0.2159, and 0.9999, respectively. The SNR, ReErr, and SSIM corresponding to RecPF method are 11.2250 dB, 0.2746, and 0.9998, respectively. From reconstructed results, it is observed that the performance of the proposed Algorithm 3 is better than RecPF.

**Figure 1:** Original image and sampling mask.

**Figure 2:** Reconstruction of Phantom.

Fig. 3 (a) and (b) show 256×256 brain image and sampling mask used in [1] with sampling ratio 33.08%. The proposed method is compared with CS-MRI method by Lustig et al. [1] (denoted as LDP). In this example, we assume μ=3. The SNR, ReErr, and SSIM values of the proposed algorithm are compared against LDP by varying the noise level from 10 to 35 and are shown in Table 1. Fig. 4 (a) and (b) show the reconstructed results by the proposed method and LDP for σ=15, and Fig. 4 (c) and (d) show the reconstructed results by the proposed method and LDP for σ=35.

The article "Removal of high density Gaussian noise in compressed sensing MRI reconstruction through modified total variation image denoising method" was retracted in 2025. Reasons: unreliable results or conclusions; concerns about the authorship.

**Figure 3:** Original image and sampling mask.

**Table 1:** SNR, ReErr, and SSIM values for the proposed method and LDP.

Noise level (*σ*)	Method	SNR (dB)	ReErr	SSIM
10	Proposed	15.4042	0.1697	0.7347
	LDP	13.9095	0.2016	0.6054

15	Proposed	13.6422	0.2079	0.6053
	LDP	11.2208	0.2748	0.4586

20	Proposed	11.5006	0.2611	0.4675
	LDP	9.1274	0.3496	0.3533

25	Proposed	9.4390	0.3373	0.3566
	LDP	7.2199	0.4355	0.2727

30	Proposed	7.7150	0.4114	0.2783
	LDP	5.6356	0.5227	0.2155

35	Proposed	6.2475	0.4871	0.2223
	LDP	4.3864	0.6035	0.1758

**Figure 4:** Reconstruction of brain MRI.

From these reconstructed results, we can see that the performance of the proposed algorithm is better than LDP.

Now let us see 220×220 chest MRI image shown in Fig. 5 (a). Fig. 5 (b) is corresponding sampling mask used in [2] with sampling ratio 38.50%. We do comparison between the proposed method and TVCMRI in [2]. Let μ=3 in Algorithm 3 and the noise deviation σ=10, the reconstructed results by the two methods are shown in Fig. 6 (a) and (b). The SNR, ReErr, and SSIM values for (a) are 17.7942 dB, 0.1289, 0.7489, respectively. The SNR, ReErr, and SSIM values for (b) are 16.0695 dB, 0.1572, 0.6794, respectively. Fig. 7 shows SNR, ReErr, and SSIM versus standard deviation *σ* between 10 and 20 for images reconstructed using the proposed method and TVCMRI. From the chart, it is observed that the proposed method yields better reconstruction results than TVCMRI does.

**Figure 5:** Original image and sampling mask.

**Figure 6:** Reconstruction of chest MRI.

**Figure 7:** Comparison between the proposed method and TVCMRI.

Finally, let us do the comparison between the proposed method and FCSA in [4]. Fig. 8 (a) shows 210×210 brain MRI image used in [4]. Fig. 8 (b) gives the sampling 44 radial lines with sampling ratio 22.60%. Let μ=3 in Algorithm 3 and the noise deviation σ=10, the reconstructed results by the two methods are shown in Fig. 9 (a) and (b). The SNR, ReErr, and SSIM values for the proposed method are 16.5932 dB, 0.1480, 0.7883, respectively. The SNR, ReErr, and SSIM values for FCSA are 15.8760 dB, 0.1608, 0.7575, respectively. Fig. 10 shows SNR, ReErr, and SSIM versus standard deviation *σ* between 10 and 30 for images reconstructed using the proposed method and FCSA. From the chart, we can see that reconstruction results for the proposed method are better than FCSA.

The article "Removal of high density Gaussian noise in compressed sensing MRI reconstruction through modified total variation image denoising method" was retracted in 2025. Reasons: unreliable results or conclusions; concerns about the authorship.

**Figure 8:** Original image and sampling mask.

**Figure 9:** Reconstruction of brain MRI.

**Figure 10:** Comparison between the proposed method and FCSA.

## 5 Conclusion

In this paper, we propose a new algorithm to remove the Gaussian noise in compressed sensing MRI reconstruction. The proposed method shows better performance in comparison with RecPF, LDR, TVCMRI, and FCSA methods in terms of SNR, Reerr, and SSIM. The performance of the algorithm has been tested at high level noise on Shepp-Logan phantom image, brain MRI images and chest MRI image. Both visual and quantitative results shows the proposed method has better denoising effectiveness than other direct reconstruction methods in CS-MRI reconstruction.

## Declarations

### Author contribution statement

Y. Zhu, W. Shen, F. Cheng, C. Jin, G. Cao: Conceived and designed the experiments; Performed the experiments; Analyzed and interpreted the data; Contributed reagents, materials, analysis tools or data; Wrote the paper.

### Funding statement

This work was supported by the National Natural Science Foundation of China (No. 11571325, No. 61772539) and the Fundamental Research Funds for the Central Universities (No. CUC2019A002, No. CUC2019B021).

### Competing interest statement

The authors declare no conflict of interest.

### Additional information

Additional Information No additional information is available for this paper.
